RETRACTED

# Study on the Oxygen Consumption Rule of Hydroponic Cotton in Different Periods

**DOI:** 10.1155/2022/4560732

**Published:** 2022-07-05

**Authors:** Yanbo Fu, Xiaojuan Rao, Qingyong Bian, Yaozu Feng, Jian Huang, Zhiguo Wang

**Affiliations:** ^1^Institute of Soil Fertilizer and Agricultural Water Saving, Xinjiang Academy of Agricultural Sciences, Urumqi, 830091, China; ^2^Xinjiang Vocational College of Agriculture, Changji, Xinjiang 831100, China; ^3^National Agricultural Experimental Station for Soil Quality Aksu, Aksu 8300914, Xinjiang, China; ^4^Science and Technology Achievements Transformation Center, Xinjiang Academy of Agricultural Sciences, Urumqi, 830091, China

## Abstract

In this paper, the decay law of dissolved oxygen in the culture solution of cotton in the seedling stage, bud stage, and blossoming and boll-forming stage was studied via hydroponic cotton experiments, and then, the oxygen consumption and its rule of cotton were explored. The results showed that with the increase of the cultivation time, the dissolved oxygen concentration of the cotton at seedling stage, bud stage, and blossoming and boll-forming stage showed an exponential function decrease. The dissolved oxygen concentration of the culture medium decreased from about 7.5 mg·L^−1^ to a relatively stable dissolved oxygen concentration, which was 4.92 mg·L^−1^, 1.64 mg·L^−1^, and 1.82 mg·L^−1^, respectively. When CK is about 7.1 mg·L^−1^, a relative equilibrium point between low oxygen absorption rate of cotton and oxygen supply is reached. The sudden drop points of the instant oxygen consumption rate of cotton seedling stage and bud stage are at about 5.15 mg·L^−1^ and 5.89 mg·L^−1^, respectively, while the sudden drop point was not obvious at the blossoming and boll-forming stage. The budding cotton can absorb oxygen when the dissolved oxygen in the culture solution is at a higher level. The blossoming and boll-forming stage cotton is more resistant to hypoxia stress.

## 1. Introduction

Oxygen is an essential nutrient factor for life activities of plants, whose growth requires sufficient oxygen supply [1]. Living cells of plants can complete their growth and metabolism at proper oxygen concentration. Unfortunately, in actual crop production, multiple factors such as flood disasters, improper irrigation, formation of root pads in substrate cultivation, or low dissolved oxygen in the nutrient solution lead to insufficient oxygen supply in the rhizosphere, resulting in hypoxia [2], which will adversely affect the growth, yield, and quality of crops, and even plant death in severe cases [3, 4] The concentration of dissolved oxygen in hydroponic culture can meet the growth needs of most plants when it reaches 4 mg·L or more [5]. It was shown that hydroponic tomato (Lycopersicon esculentum) produced oxygen deficiency symptoms when the dissolved oxygen content of the nutrient solution is less than 3 mg [6]. When the O_2_ supply of the root system is insufficient, the respiration of the root is only 1/3 of the normal condition [7]. The hypoxia signal produced by the root will be transmitted to the crown, slowing the absorption and transmission of growth information, including water, nutrient ions, and plant auxins [8] which slowed down plant growth. Root respiration is the energy source for root metabolic activity and directly controls the growth of surface crops [9]. The energy consumed by roots to absorb water and nutrients is mainly supplied by root aerobic respiration ([10–12]; ). Many researchers [13–15] have also reported that hypoxia in the root zone of crops restricts root development and plant growth. Hypoxia in the rhizosphere seriously restricts the growth of crops. It has gradually become a hot spot to explore the effects of aerobic measures on plant growth and the promotion of increased oxygen content on crop yields. At the same time, more scholars have set to explore the physiological and biochemical responses and molecular mechanisms of plants to hypoxic environments. Therefore, the study on the response and adaptation mechanism of crops to changes in rhizosphere oxygen content is of great significance to crop aerobic irrigation technology and breeding. In this paper, hydroponic cotton as the research object, the oxygen consumption rule of cotton was studied by monitoring the change of dissolved oxygen in the culture solution of cotton in different periods, thus providing theoretical data-based support for the research of aeration technology.

RETRACTED

## 2. Materials and Methods

### 2.1. Experiment Materials

The tested cotton was Xinluzao 41. The hydroponic test was carried out in the network room of the National Grey Desert Soil Test Station of Anningqu Test Site in Urumqi, Xinjiang. The size of the petri dish was 50 × 38 × 23 cm, the solution volume was 20 L, and each pot had 6 cotton plant. The nutrient solution was composed of Hoagland's complete nutrient solution and Anon micronutrient solution, with a pH of about 6.5.

### 2.2. Basic Information of the Experiment

On June 16, 2019, the seedlings were cultivated on sand in the incubator with intelligent light, and on June 25, 2019, the seedlings were cultivated in a petri dish. Each pot had 6 cotton seedlings, and the size of the petri dish was 50 × 38 × 23 cm, and the nutrient solution volume was 20 L. After transplanting, the nutrient solution is replaced every 10 days. Blow into the petri dish every 6 hours for 30 minutes.

During the three periods of July 5th (seedling stage), August 14th (bud stage), and September 24th (blossoming and boll-forming stage), cotton plants with the same growth rate were selected and transplanted into petri dishes with the same dissolved oxygen concentration. The oxygen consumption of cotton was then monitored. Two treatments were set up, that is, blank CK-untransplanted cotton and hydroponic cotton CO-transplant 6 cotton with same growth rate. Each treatment was done for 3 times.

### 2.3. Detection Methods

#### 2.3.1. Observation and Investigation

The dissolved oxygen concentration in the nutrient solution of cotton was measured dynamically and continuously during the cultivation period. After the dissolved oxygen concentration was stable after increasing oxygen, cotton was transplanted on July 5 (seedling stage), August 14 (bud stage), and September 24, (blossoming and boll-forming stage), respectively, and the change of dissolved oxygen in the culture medium was monitored in time until the dissolved oxygen in the culture medium decreased to a relatively stable level.

#### 2.3.2. Analysis and Measurement Methods

The dissolved oxygen was determined by YSI5000 (YSI Company of the United States), which bears the function of automatic temperature compensation with an agitator. The concentration of dissolved oxygen in the petri dish was measured periodically, and the specific parameters were calculated as follows: the change of dissolved oxygen concentration in petri dish-the difference of the monitoring value of dissolved oxygen in solution per unit time; the decay rate of dissolved oxygen in solution-the change of dissolved oxygen concentration in petri dish/time; and oxygen consumption rate per plant − decay rate of dissolved oxygen in solution × volume/plant number.

### 2.4. Statistical Analysis

WPS Excel software was used for data processing, and DPS 9.05 software was adopted for statistical analysis.

## 3. Result Analysis

### 3.1. Changes in the Content of Dissolved Oxygen in the Culture Fluid

The changes of dissolved oxygen concentration (DO) in the control check (CK) and hydroponic cotton (CO) were dynamically and continuously monitored on July 5^th^ (seedling stage), August 14 (bud stage), and September 24th (blossoming and boll-forming stage), respectively, until the dissolved oxygen concentration in the culture medium decreased to a relatively stable level. As shown in Figure 1, the concentration of dissolved oxygen in the culture medium of hydroponic cotton at the seedling stage (Figure 1(a)) decreased from 7.75 mg·L^−1^ to 4.92 mg·L^−1^ 16 hours later, decreased by 2.83 units and 36.5%. The dissolved oxygen concentration of CK decreased from 7.75 mg·L^−1^ to 7.09 mg·L^−1^, decreased by 0.66 units and 8.5%. 11 hours later, the concentration of dissolved oxygen in the culture medium of hydroponic cotton at bud stage (Figure 1(b)) decreased from 7.38 mg·L^−1^ to 1.64 mg·L^−1^, decreased by 5.74 units and 77.8%. The concentration of dissolved oxygen in CK decreased from 7.75 mg·L^−1^ to 7.12 mg·L^−1^, decreased by 0.63 units and 8.1%. After 10-hour culture, the concentration of dissolved oxygen of culture medium at the blossoming and boll-forming stage (Figure 1(c)) dropped from 7.62 mg·L^−1^ to 1.82 mg·L^−1^, decreased by 5.80 units and 76.1%. The concentration of dissolved oxygen in blank CK decreased by 0.62 units or 8.0%, from 7.75 mg·L^−1^ to 7.13 mg·L^−1^. The dissolved oxygen concentration of the hydroponic cotton culture solution decreases exponentially with the increase of culture time. Dissolved oxygen content decreased trend: seedling stage < bud stage < blossoming and boll − forming stage. The decay variables when the dissolved oxygen of the culture fluid was reduced to a relatively stable level were as follows: CK (0.62 − 0.66 mg · L^−1^) < seedling stage (2.17 mg · L^−1^) < bud stage (5.11 mg · L^−1^) < blossoming and boll − forming stage (5.18 mg·L^−1^). The dissolved oxygen concentration in CK culture medium decreased by about 8%. The changes in dissolved oxygen in CK was 23.3% of the change in dissolved oxygen in CO AT seedling stage and about 10% of the change in dissolved oxygen in CO at bud stage and blossoming and boll-forming stage, which affects the value of cotton oxygen consumption and needs to be corrected for dissolved oxygen.

RETRACTED

### 3.2. Oxygen Consumption per Cotton Plant

The changes of dissolved oxygen in the culture solution were observed, and the oxygen consumption and simulated value of a single cotton plant were analyzed in the three growth stages during the monitoring period. As shown in Figure 2, when the dissolved oxygen of the culture fluid drops to a relatively stable level, the oxygen consumption of a single cotton plant increases from 0.73 mg to 7.23 mg after 16 hours of culture of cotton in the seedling stage (Figure 2(a)). After the budding cotton (Figure 2(b)) was cultivated for 11 hours, its oxygen consumption per plant increased from 5.93 mg to 17.03 mg. After cultivating blossoming and boll-forming stage cotton (Figure 2(c)) for 10 hours, the oxygen consumption of individual cotton increased from 1.17 mg to 17.27 mg. As the dissolved oxygen in the culture fluid dropped to a relatively stable level, single cotton in the seedling stage consumes the least oxygen (7.23 mg), followed by that at the bud stage (17.03 mg) and the blossoming and boll-forming stage (17.27 mg).

RETRACTED

The oxygen consumption models of the cotton at seedling stage, bud stage, and blossoming and boll-forming stage are *y* = 0.0041*x*^2^ + 0.4375*x* − 0.4054 (*R*^2^ = 0.9697), *y* = −0.0622*x*^2^ + 1.9241*x* + 3.5237 (*R*^2^ = 0.9984), and *y* = −0.0819*x*^2^ + 2.4565*x* + 0.7518 (*R*^2^ = 0.9984), respectively. The oxygen consumption per cotton plant was simulated at 2 h, 4 h, 6 h, 8 h, 10 h, and 12 h using the oxygen consumption model, and specific values were summarized in Table 1. When simulated at 12 hours, the oxygen consumption per plant of cotton was the highest in the blossoming and boll-forming stage (18.44 mg), followed by the bud stage (17.66 mg) and seedling stage (4.25 mg). The oxygen consumption at the bud stage before 7.05 h was greater than that of the blossoming and boll-forming stage, and the opposite trend appeared after 7.05 h, indicating that the oxygen absorption capacity of the cotton at blossoming and boll-forming stage at low oxygen concentrations was higher than that of the bud stage.

### 3.3. Oxygen Consumption Rate per Cotton Plant

By observing the dissolved oxygen in the culture solution, the cotton oxygen consumption rate, the instant oxygen consumption rate, and the simulation value of a single cotton were analyzed in the seedling stage, bud stage, and blossoming and boll-forming stage. As shown in Table 2, the oxygen consumption rate at the seedling stage fluctuates between 0.32 mg·h^−1^ and 0.51 mg·h^−1^, and its immediate oxygen consumption rate ranges from 0.27 mg·h^−1^ to 0.80 mg·h^−1^. The oxygen consumption rate and instant oxygen consumption rate of cotton at the bud stage decreased in a power function trend; the oxygen consumption rate decreased from 4.75 mg·h^−1^ to 1.55 mg·h^−1^, decreased by 3.20 units and 67.4%. The immediate oxygen consumption rate was reduced from 4.75 mg·h^−1^ to 0.52 mg·h^−1^, reduced by 4.23 units and 89.1%. The oxygen consumption rate and instant oxygen consumption rate at the blossoming and boll-forming stage decreased in a power function trend. The oxygen consumption rate decreased from 3.5 mg·h^−1^ to 1.73 mg·h^−1^, reduced by 1.77 units and 50.7%. The immediate oxygen consumption rate was reduced from 3.1 mg·h^−1^ to 1.12 mg·h^−1^, reduced by 2.38 units and 68.1%. The above analyses showed that the oxygen consumption rate and instant oxygen consumption rate of cotton at the seedling stage indicated no obvious changes, which may be due to lower oxygen consumption of seedling stage cotton and the dissolved oxygen greatly affected by the environment.

As shown in Table 3, the models for instant oxygen consumption rate of cotton at the bud stage and blossoming and boll-forming stage are *y* = 5.4839*x*^−0.859^ (*R*^2^ = 0.8934) and *y* = 2.7004*x*^−0.35^ (*R*^2^ = 0.8762), respectively. This model was used to simulate the instant oxygen consumption rate at 0.5 h, 1 h, 2 h, 4 h, 6 h, 8 h, and 12 h. The instant oxygen consumption rate of the bud stage is reduced from 9.95 mg·h^−1^ to 0.65 mg·h^−1^, reduced by 9.30 units, with a decrease of 93.5%. The immediate oxygen consumption rate of the blossoming and boll-forming stage was reduced from 2.70 mg·h^−1^ to 1.13 mg·h^−1^, and the oxygen consumption rate was reduced by 2.31 units, with a decrease of 67.1%. The oxygen consumption rate of the budding cotton before 4 h is greater than that of the blossoming and boll-forming stage. After 4.03 h, the oxygen consumption rate of the cotton bud stage is less than that of the blossoming and boll-forming stage. At this time, the dissolved oxygen concentration of the bud stage and the blossoming and boll-forming stage was 4.04 mg·h^−1^ and 4.42 mg·h^−1^, respectively. Furthermore, when the dissolved oxygen concentration of the culture fluid reaches a high level, the oxygen absorption capacity of cotton in the bud stage is better than that of the blossoming and boll-forming stage, while as dissolved oxygen concentration arrives at a low level, the cotton at the bud stage absorbs less oxygen than that at the blossoming and boll-forming stage. The oxygen consumption rate of stage and bud stage cotton is greatly depending on the dissolved oxygen concentration of the culture solution.

RETRACTED

### 3.4. Relationship between Dissolved Oxygen Concentration and Oxygen Consumption Rate of Single Cotton Plant

As shown in Figure 3, the cotton at the seedling stage (Figure 3(a)) has no significant functional relationship between the dissolved oxygen concentration of the culture medium and the instant oxygen consumption rate of cotton. When the dissolved oxygen concentration reaches at 5.11 mg·L^−1^, there is a sudden jump in the instant oxygen consumption rate, indicating that cotton is sensitive to the dissolved oxygen concentration of the culture solution during the seedling stage, and the oxygen absorption rate of cotton will drop rapidly if the dissolved oxygen concentration of the culture solution is lower than 5.11 mg·L^−1^. The dissolved oxygen concentration in the culture solution of the bud stage and blossoming and boll-forming stage (Figure 3(b)) of cotton demonstrated a quadratic function relationship with the instantaneous oxygen consumption rate of cotton, and the instant oxygen consumption rate model of bud stage and blossoming and boll-forming stage cotton was *y* = 0.2422*x*^2^ − 1.2491*x* + 2.3975 (*R*^2^ = 0.9004) and *y* = 0.114*x*^2^ − 0.673*x* + 2.2177 (*R*^2^ = 0.9212), respectively. When the dissolved oxygen concentration of bud stage cotton reaches 5.89 mg·L^−1^, the immediate oxygen consumption rate jumps, informing that bud stage cotton is sensitive to the dissolved oxygen concentration of the culture solution. The instantaneous oxygen consumption rate of cotton was simulated using the quadratic function model when the dissolved oxygen concentration of the culture solution arrived at 2 mg·L^−1^, 4 mg·L^−1^, 6 mg·L^−1^, 7 mg·L^−1^, and 8 mg·L^−1^, respectively. The instantaneous oxygen consumption rate of cotton at the seedling stage was 0.54-0.69 mg·h^−1^, increased from 0.87 mg·h^−1^ to 7.91 mg·h^−1^ at the bud stage, and elevated from 1.33 mg·h^−1^ to 4.13 mg·h-1 at the blossoming and boll-forming stage. When the dissolved oxygen concentration is 4.15 mg·L^−1^, the instant oxygen consumption rate at the bud stage is equal to that at blossoming and boll-forming stage, and when the dissolved oxygen concentration is less than 4.15 mg·L^−1^, the instant oxygen consumption rate at the bud stage is less than that at the blossoming and boll-forming stage. Collectively, it was indicated that the blossoming and boll-forming stage cotton was less affected by the concentration of dissolved oxygen, and thus, the resistance to stress of cotton was improved (see Table 4).

RETRACTED

## 4. Results

The dissolved oxygen concentration of the hydroponic culture solution for cotton decreases exponentially with the increase of the culture time. The cotton at the blossoming and boll-forming stage has the largest reduction in dissolved oxygen content, followed by the bud stage and seedling stage. The time for the dissolved oxygen in the culture solution to decrease to a relatively stable level is 16 h at the seedling stage, 11 h at the bud stage, and 10 h at the blossoming and boll-forming stage, and the decay variable CK (0.62 − 0.66 mg · L^−1^) < seedling stage (2.17 mg · L^−1^) < bud stage (5.11 mg · L^−1^) < blossoming and boll − forming stage (5.18 mg·L^−1^).

When the dissolved oxygen in the culture fluid drops to a relatively stable level, the oxygen consumption per cotton plant is seedling stage (7.23 mg) < bud stage (17.03 mg) < blossoming and boll − forming stage (17.27 mg). The oxygen consumption models per plant at seedling stage, bud stage, and blossoming and boll-forming stage were *y* = 0.0041*x*^2^ + 0.4375*x* − 0.4054 (*R*^2^ = 0.9697), *y* = −0.0622*x*^2^ + 1.9241*x* + 3.5237 (*R*^2^ = 0.9984), and *y* = −0.0819*x*^2^ + 2.4565*x* + 0.7518 (*R*^2^ = 0.9984), respectively. The instant oxygen consumption rate of single plant at the seedling stage fluctuates between 0.27 mg·h^−1^ and 0.80 mg·h^−1^, and the instant oxygen consumption rate models of cotton at the bud stage and blossoming and boll-forming stage were *y* = 5.4839*x*^−0.859^ (*R*^2^ = 0.8934) and *y* = 2.7004*x*^−0.35^ (*R*^2^ = 0.8762), respectively.

RETRACTED

With the increase of dissolved oxygen concentration in culture medium, the immediate oxygen consumption rate of cotton at the bud stage and blossoming and boll-forming stage increased with a quadratic function. When the dissolved oxygen concentration of the culture fluid ranges from 2 to 8 mg·L^−1^, the instant oxygen consumption rate at the seedling stage, bud stage, and blossoming and boll-forming stage cotton is 0.87-7.91 mg·h^−1^ and 1.33-6.89 mg·h^−1^, respectively, and the immediate oxygen consumption rate of seedling stage cotton is initially determined to be about 0.54-0.69 mg·h^−1^, indicating that the oxygen concentration exerts a significant effect on the oxygen consumption rate of cotton. The results of this study provide a theoretical basis for the fine quantitative study of cotton oxygen demand in future.

## 5. Discussion

### 5.1. Dissolved Oxygen in Culture Solution

Dissolved oxygen in water mainly comes from atmospheric oxygen. The saturation value of dissolved oxygen in natural water is 9 mg·L^−1^, and the amount of dissolved oxygen in water at room temperature is about 7-14 mg·L^−1^ [16]. The dissolved oxygen in the soil solution generally ranges from 4.70 to 5.44 mg·L^−1^. The content of dissolved oxygen in water is related to multiple factors, such as changes in meteorological parameters, water temperature, water depth, and solutes in water [17–23]. When the consumption rate of dissolved oxygen is greater than the rate of oxygen dissolving into water, the content of dissolved oxygen will approach to zero. In this study, the dissolved oxygen concentration of the culture solution was about 7.5 mg·L^−1^, and the dissolved oxygen concentration of each treatment culture solution fell to a relatively stable level. In detail, the dissolved oxygen concentration at seedling stage was 4.92 mg·L^−1^, 1.64 mg·L^−1^ at ^the^ bud stage and 1.82 mg·L^−1^ at the blossoming and boll-forming stage. At this time, it is possible to reach a balance point between oxygen consumption and oxygen supply. Seedling stage cotton and budding cotton show a rapid decrease in oxygen consumption rate at about 5.15 mg·L^−1^ and at 5.89 mg·L^−1^, while blossoming and boll-forming stage cotton exhibited no significant drop point [24].

### 5.2. Cotton Oxygen Consumption Rule

Cotton is a crop sensitive to low oxygen environment [24]. The dissolved oxygen and oxygen consumption in culture medium were different in different culture time. When the concentration of dissolved oxygen decreased to 2.79 ± 0.11 mg·L^−1^ at 7.05 h, the oxygen consumption of cotton at bud stage was equal to that at the blossoming and boll-forming stage, and when the concentration of dissolved oxygen decreased to 3.01 ± 0.12 mg·L^−1^ at 6.5 h, the oxygen consumption rates of cotton at the bud stage were equivalent to those at the blossoming and boll-forming stage. When the dissolved oxygen concentration drops to 4.23 ± 0.19 mg·L^−1^ when cultured for 4.03 h, the instant oxygen consumption rate at the bud stage was equal to the blossoming and boll-forming stage, and after that time point, the oxygen consumption at the bud stage was smaller than the blossoming and boll-forming stage, indicating that the budding cotton has a higher oxygen absorption capacity under higher dissolved oxygen concentration than the blossoming and boll-forming stage, and the blossoming, and boll-forming stage cotton has higher oxygen absorption capacity under low oxygen concentration, indicating that the cotton at the bud stage is more sensitive to dissolved oxygen concentration. During the seedling stage, cotton is sensitive to oxygen concentration due to its lack of roots and weak oxygen absorption capacity. The dissolved oxygen in the culture solution must reach around 5.15 mg·L^−1^ to maintain the higher oxygen consumption rate of seedling cotton. The dissolved oxygen of the culture solution must exceed 5.89 mg·L^−1^ to ensure the higher oxygen consumption rate of budding cotton.

RETRACTED

## 6. Conclusion

For the hydroponic cotton, the dissolved oxygen concentration of culture solution decreases exponentially with the increase of the cultivation time, and the dissolved oxygen content showed the greatest decrease in the blossoming and boll-forming stage, followed by the bud stage and the seedling stage. When the dissolved oxygen concentration is 5.11 mg·L^−1^, seedling cotton has a sudden jump in oxygen consumption rate. When the dissolved oxygen concentration is 5.89 mg·L^−1^, budding cotton exhibits a sudden jump in oxygen consumption rate, indicating that seedling cotton is more sensitive to the dissolved oxygen concentration of the culture fluid than the budding cotton. When the dissolved oxygen concentration is less than 4.15 mg·L^−1^, the immediate oxygen consumption rate at the bud stage is less than that of the blossoming and boll-forming stage, and the oxygen absorption capacity of the bud stage is lower than that of the blossoming and boll-forming stage. The dissolved oxygen concentration of the culture solution is higher than 4.15 mg·L^−1^, the immediate oxygen consumption rate of the cotton at bud stage is greater than that at the blossoming and boll-forming stage, and the oxygen absorption capacity is higher than that of the blossoming and boll-forming stage, indicating that the cotton bud stage cotton oxygen consumption rate is greatly affected by the dissolved oxygen concentration of the culture solution. The cotton at the blossoming and boll-forming stage is less affected by the concentration of dissolved oxygen. To sum up, cotton is sensitive to oxygen and hypoxia, and the rate of absorbing oxygen is significantly depending on the concentration of dissolved oxygen (influence degree is seedling stage > bud stage > blossoming and boll − forming stage). The oxygen uptake ability of budding cotton was higher than that of the blossoming and boll-forming stage, and cotton at the blossoming and boll-forming stage cotton has strong resistance to hypoxia. When the dissolved oxygen in the culture medium is higher, the oxygen uptake capacity of cotton is higher than that of the blossoming and boll-forming stage cotton.

RETRACTED

## Figures and Tables

**Figure 1:** Changes of dissolved oxygen in culture medium in different periods (mg·L^−1^).

**Figure 2:** Oxygen consumption per cotton plant in different periods (mg).

**Figure 3:** Changes of oxygen consumption rate of cotton in different periods.

**Table 1:** Simulation table of oxygen consumption per cotton plant.

Growth period	The oxygen consumption model	*R* ^2^	The oxygen consumption was simulated at different incubation periods (mg)					
			2 h	4 h	6 h	8 h	10 h	12 h
Seedling period	*y* = 0.0041*x*^2^ + 0.4375*x* − 0.4054	0.9697	0.45	1.28	2.07	2.83	3.56	4.25
Budding period	*y* = −0.0622*x*^2^ + 1.9241*x* + 3.5237	0.9984	7.12	10.22	12.83	14.94	16.54	17.66
Flowering and boll period	*y* = −0.0819*x*^2^ + 2.4565*x* + 0.7518	0.9984	5.34	9.27	12.54	15.16	17.13	18.44

**Table 2:** Statistical data of oxygen consumption rate per cotton plant in different periods.

Growth period	Parameter	Value					
Seedling period	*T* (h)	2.00	4.00	8.00	11.00	13.00	16.00
	Rate of decay of DO (mg·h^−1^)	0.37	0.32	0.34	0.47	0.51	0.45
	Rate of immediate decay of DO (mg·h^−1^)	0.37	0.27	0.37	0.80	0.77	0.19
Budding period	*T* (h)	1.25	3.25	5.67	7.00	9.00	11.00
	Rate of decay of DO (mg·h^−1^)	4.75	2.77	2.16	2.01	1.78	1.55
	Rate of immediate decay of DO (mg·h^−1^)	4.75	1.53	1.34	1.40	0.95	0.52
Flowering and boll period	*T* (h)	0.75	1.92	4.80	5.88	7.85	10.00
	Rate of decay of DO (mg·h^−1^)	3.47	2.80	2.20	2.07	1.89	1.73
	Rate of immediate decay of DO (mg·h^−1^)	3.44	2.24	1.74	1.48	1.37	1.12

**Table 3:** Simulation table of instantaneous oxygen consumption rate per cotton plant.

Growth period	Immediate oxygen consumption rate model	*R* ^2^	Simulation value (mg·h^−1^)						
			0.5 h	1 h	2 h	4 h	6 h	8 h	12 h
Budding period	*y* = 5.4839*x*^−0.859^	0.8934	9.95	5.48	3.02	1.67	1.18	0.92	0.65
Flowering and boll period	*y* = 2.7004*x*^−0.35^	0.8762	3.44	2.70	2.12	1.66	1.44	1.30	1.13

RETRACTED

**Table 4:** Simulation table of immediate oxygen consumption rate per cotton plant.

Growth period	Relationship model between dissolved oxygen concentration and cotton oxygen consumption rate	*R* ^2^	Simulation value (mg·h^**-1**^)					
			Set the DO (mg·h^−1^)					
			2	4	6	7	8	10
Seedling period	*y* = −0.2528*x*^2^ + 3.1394*x* − 9.0415	0.5079	-3.77	-0.53	0.69	0.54	-0.11	-2.93
Budding period	*y* = 0.2422*x*^2^ − 1.2491*x* + 2.3975	0.9004	0.87	1.28	3.62	5.52	7.91	14.13
Flowering and boll period	*y* = 0.114*x*^2^ − 0.673*x* + 2.2177	0.9212	1.33	1.35	2.28	3.09	4.13	6.89

## Data Availability

The dataset used in this paper is available from the corresponding author upon request.
